# Mathematical Modeling Investigation of Violence and Racism Coexistence as a Contagious Disease Dynamics in a Community

**DOI:** 10.1155/2022/7192795

**Published:** 2022-07-26

**Authors:** Shewafera Wondimagegnhu Teklu, Birhanu Baye Terefe

**Affiliations:** Department of Mathematics, Collage of Natural and Computational Sciences, Debre Berhan University, Debre Berhan, Ethiopia

## Abstract

Recently, violence, racism, and their coexistence have been very common issues in most nations in the world. In this newly social science discipline mathematical modelling approach study, we developed and examined a new violence and racism coexistence mathematical model with eight distinct classes of human population (susceptible, violence infected, negotiated, racist, violence-racism coinfected, recuperated against violence, recuperated against racism, and recuperated against the coinfection). The model takes into account the possible controlling strategies of violence-racism coinfection. All the submodels and the violence-racism coexistence model equilibrium points are calculated, and their stabilities are analyzed. The model threshold values are derived. As a result of the model qualitative analysis, the violence-racism coinfection spreads under control if the corresponding basic reproduction number is less than unity, and it propagates through the community if this number exceeds unity. Moreover, the sensitivity analysis of the parameter values of the full model is illustrated. We have applied MATLAB ode45 solver to illustrate the numerical results of the model. Finally, from qualitative analysis and numerical solutions, we obtain relevant and consistent results.

## 1. Introduction

The World Health Organization defines violence as “the intentional use of physical force or power, threatened or actual, against oneself, against another person or against a group or community, which either results in or has a high likelihood of resulting in injury, death, psychological harm mal-development, or deprivation.” It is considered as a common universal public health issue due to its frequency and consequences against community [1]. Ethnic violence is a comprehensive term for violence that is prompted from hatred or racism or ethnic stresses or ethnic conflict [2]. Violence against females occurs in all types of society almost in the entire world and affects girls and women of all ages and in all stages of life. In western countries, it has not been until quite recently (1979) that the intimate violence partner was institutionally identified and condemned, and its origin is found in feminists in the 1950s [3].

Globalization and migration flows induce a rapidly enhancing of ethnic and racism diverseness within many nations in the world [4]. The spreading of racism in a mixed culturally diverse society affects in a significant manner in all aspects of their life. The widespread proliferation of racism can lead to a series of serious hazards, such as social instability, impacts on election results, or large financial losses. It can be considered as mind infection, and its expansion and impact on individuals indicted similar to infectious diseases, like tuberculosis (TB), COVID-19, and pneumonia pathogenic agents [5]. Various social science studies related to individual behaviors such as violence, racism, social media addiction, and corruption have been carried out by many scholars throughout the world [6–15]. Violence and violation are crucially at the heart of racism, and hence, in principle, the coexistence of violence and racism on individuals in a community is assured [14].

Any situation, such as individuals' behavior that can be spreading from human being to human being, can lead to similar unstable epidemiological infectious disease conditions. Indeed, there are a lot of literatures associated with the happening of behavioral contagion related to individuals' mental health situation. Violence is one condition in which behavioral contagion may happen, and some contagious behaviors have been observed to occur in situations of higher density and in larger groups, consistent with the behavior of infectious epidemics [16].

Mathematical modeling has a continuous fundamental role in understanding of the various aspects of dynamical system of real-world situations like [17–21]. It has been formulated and analyzed in different disciplines such as natural sciences as well as social science like [1–5, 9, 22–33]. Many researchers have applied infectious disease dynamics model to violence, racism, social media addition, corruption, and other social situations. From those researchers, some were applied modeling for social media addiction [34], some were used modeling for violence [1–3, 33], some were applied modeling for racism [4, 5, 25], and others used modeling for corruption dynamics [22–24, 26–28, 35–38]. However, to the best of our knowledge, no one has developed and analyzed a mathematical model on violence-racism coexistence on individuals in a given society. Therefore, in this newly proposed violence-racism coexistence model, we are motivated and interested in filling the specified gap, and we attempt to examine this connection by constructing a mathematical model of violence-racism coexistence contagion with controlling strategies.

The remaining part of this study is organized as follows. In Section 2, we describe and formulate the compartmental mathematical model of violence-racism coexistence. In Section 3, we analyzed the submodels and the main model. We determined the equilibrium points and basic reproduction numbers and analyzed stabilities of the submodels and the main model equilibrium points. In Section 4, we have carried out the sensitivity analysis and numerical simulations. Finally, we have performed discussions and conclusions in Section 5.

## 2. Violence and Racism Coexistence Model Formulation

In this study, we considered both violence and racism as chronic contagious diseases, and we divide the total number of human population *N*(*t*) in a given time *t* into eight mutually exclusive social states. Those are susceptible for either violence or racism *S*(*t*), violence infected *V*(*t*), negotiated *U*(*t*), recuperated from violence *R*_1_(*t*), racism infected *R*(*t*), recuperated from racism *R*_2_(*t*), violence and racism coinfected *I*_*vr*_(*t*), and recuperated from coinfected *R*_3_(*t*) such that *N*(*t*) = *S*(*t*) + *V*(*t*) + *U*(*t*) + *R*_1_(*t*) + *R*(*t*) + *R*_2_(*t*) + *I*_*vr*_(*t*) + *R*_3_(*t*).

### 2.1. Description of Social State Variables of the Model

- Susceptible individuals for both violence and racism are those group of people who are at risk of violence and racism. These individuals have not received, heard, or acted violence and racism spreading activities described by *S*(*t*)
- Violence-infected individuals are those group of people who use physical force to harm, injure, damage, or destroy someone to spreading violence described by *V*(*t*)
- Negotiated individuals are the group of individuals who are ongoing to reach an agreement with a formal discussion between people described by *U*(*t*)
- Recuperated from violence is a group of individuals who made compatible, consistent, or group to become friendly again after an argument described by *R*_1_(*t*)
- Racism-infected is the group of individuals who have received or heard racist information and support the racist activity. These people are actively spreading the racist ideology and described by *R*(*t*)
- Recuperated from racism is a group of individuals who reject the racist ideology by *R*_2_(*t*)
- Violence and racism coinfected is a group of individuals who are infected by both violence and racism described by *I*_*vr*_(*t*)
- Recuperated from coinfected is a group of individuals who made compatible, consistent, or group to become friend again and reject the racist ideology described by *R*_3_(*t*)

### 2.2. Basic Assumptions of the Model

- Coinfected individuals can transmit violence and racism infections one after the other and do not transmit simultaneously
- Individuals acquire violence infection following effective contacts with people infected with violence (*V* and *I*_*vr*_ classes) at the force of infection rate given by

(1) $$\begin{array}{c} \lambda_{v}=\beta_{1}\left(V+\theta_{2}I_{vr}\right) \end{array}$$

(iii) Individuals acquire racism infection from (*R* and *I*_*vr*_ classes) at the force of infection rate given by

(2) $$\begin{array}{c} \lambda_{r}=\beta_{2}\left(R+\theta_{1}I_{vr}\right) \end{array}$$

(iv) Human population is variable and homogeneous
(v) We did not consider racism only controlling mechanisms for the coinfectious individuals in the community, and we used coinfection instead of behavior coexistence

### 2.3. Description of Model Parameters Is Given in Table 1

Using the model assumptions and the flow diagram of violence and racism coexistence transmission dynamics given in Figure 1, the corresponding dynamical system is given by

(3) $$\begin{array}{c} \frac{dS}{dt}=\Lambda +\alpha R_{1}+\rho R_{2}+\theta R_{3}–\left(\lambda_{v}+\lambda_{r}+\mu \right)S,\\ \frac{dV}{dt}=\lambda_{v}S–\left(\delta +\kappa \lambda_{r}+\mu \right)V,\\ \frac{dU}{dt}=\delta V–\left(\varepsilon +\mu \right)U,\\ \frac{dR}{dt}=\lambda_{r}S+\omega I_{vr}-\left(\sigma +\beta \lambda_{v}+\mu \right)R,\\ \frac{dI_{vr}}{dt}=\beta \lambda_{v}R+\kappa \lambda_{r}V-\left(\phi +\omega +\mu \right)I_{vr},\\ \frac{dR_{1}}{dt}=\varepsilon U–\left(\alpha +\mu \right)R_{1},\\ \frac{dR_{2}}{dt}=\sigma R-\left(\rho +\mu \right)R_{2},\\ \frac{dR_{3}}{dt}=\phi I_{vr}-\left(\theta +\mu \right)R_{3}. \end{array}$$

### 2.4. Basic Properties of the Coexistence Model

Since the violence-racism coexistence model (3) deals with human population which cannot be negative, we need to show that all the solutions of system (3) remain positive with positive initial conditions in the bounded region

(4) $$\begin{array}{c} \Omega =\left\{\left(S,V,U,R,I_{vr},R_{1},R_{2},R_{3}\right)\in {\mathbb{R}}_{+}^{8},N\leq \frac{\Lambda }{\mu }\right\}. \end{array}$$

**Theorem 1 .**

Let  *S*(0) > 0, *V*(0) > 0, *U*(0) > 0, *R*_1_(0) > 0, *R*(0) > 0, *R*_2_(0) > 0, *I*_*vr*_(0) > 0, and *R*_3_(0) > 0 be the initial solutions of the model (3); then, *S*(*t*), *V*(*t*), *U*(*t*),*R*_1_(*t*), *R*(*t*), *R*_2_(*t*),  *I*_*vr*_(*t*), and *R*_3_(*t*) are positive in ℝ_+_^8^ for all time *t* > 0.

**Proof**

Let us define *τ* = sup{*t* > 0 : *S* (t) > 0, *V*(*t*) > 0, *U*(*t*) > 0, *R*(*t*) > 0, *I*_*vr*_(*t*) > 0, *R*_1_(*t*) > 0, *R*_2_(*t*) > 0, *R*_3_(*t*) > 0}.

Since *S*(*t*), *V*(*t*), *U*(*t*), *R*(*t*), *I*_*vr*_(*t*), *R*_1_(*t*), *R*_2_(*t*), and *R*_3_(*t*)  are continuous, we deduce that *τ* > 0. If *τ* = +∞, then positivity holds, but, if 0 < *τ* < +∞, *S*(*τ*) = 0 or *V*(*τ*) = 0 or *U* (*τ*) = 0 or *R*(*τ*) = 0 or *I*_*vr*_( *τ* ) = 0 or *I*_*vr*_(*τ*) = 0, *R*_1_(*τ*) = 0 or *R*_2_(*τ*) = 0, or *R*_3_(*τ*) = 0.

Here, from the first equation of the model differential equation in (3), we do have

(5) $$\begin{array}{c} \frac{dS}{dt}+\left(\lambda_{v}+\lambda_{r}+\mu \right)S=\Lambda +\alpha R_{1}+\rho R_{2}+\theta R_{3}. \end{array}$$

Then, by integrating using the method of integrating factor, we got

(6) $$\begin{array}{c} S\left(\tau \right)=M_{1}S\left(0\right)+M_{1}\int_{0}^{\tau }\exp^{\int \left.\left(\lambda_{v}\left(t\right)+\lambda_{r}\left(t\right)+\mu \right)\right)dt}\left(\Lambda +\alpha R_{1}\left(t\right)+\rho R_{2}\left(t\right)+\theta R_{3}\left(t\right)\right)dt>0, \end{array}$$

where *M*_1_ = exp^−(*μτ* + ∫_0_^*τ*^(*λ*_*v*_(*w*) + *λ*_*r*_(*w*))^ > 0, *S*(0) > 0, and from the definition of *τ*, we have *R*_1_(*t*) > 0, *R*_2_(*t*) > 0, *R*_3_(*t*) > , then the solution *S*(*τ*) > 0 and hence *S*(*τ*) ≠ 0.

Again, from the second equation of the model differential equation in (3), we do have

(7) $$\begin{array}{c} \frac{dV}{dt}+\left(\delta +\kappa \lambda_{r}+\mu \right)V=\lambda_{v}S, \end{array}$$

and we have obtained *S*(*τ*) = *M*_1_*S*(0) + *M*_1_∫_0_^*τ*^exp^∫(*δ* + *κλ*_*r*_ + *μ*)*dt*^(*λ*_*v*_*S*)*dt* > 0,where *M*_1_ = exp^−(*μτ* + *δτ* + ∫_0_^*τ*^(*κλ*_*r*_(*w*))^ > 0, *S*(0) > 0, and from the definition of *τ*, the solution *S*(*τ*) > 0; hence, *S*(*τ*) ≠ 0.

Similarly, *V*(*τ*) > 0; hence, *V*(*τ*) ≠ 0; *U*(*τ*) > 0; hence, *U*(*τ*) ≠ 0; *R*(*τ*) > 0; hence, *R*(*τ*) ≠ 0; *R*_1_(*τ*) > 0; hence, *R*_1_(*τ*) ≠ 0; *R*_2_(*τ*) > 0; hence, *R*_2_(*τ*) ≠ 0; and *R*_3_(*τ*) > 0; hence, *R*_3_(*τ*) ≠ 0.

Thus, based on the definition, *τ* is not finite which means *τ* = +∞, and hence, all the solutions of the system (3) are nonnegative.

**Theorem 2 .**

The region *Ω* in system (4) is bounded in the space ℝ_+_^8^.

**Proof**

The total number of human populations *N*(*t*) is

(8) $$\begin{array}{c} N\left(t\right)=S\left(t\right)+V\left(t\right)+U\left(t\right)+R_{1}\left(t\right)+R\left(t\right)+R_{2}\left(t\right)+I_{vr}\left(t\right)+R_{3}\left(t\right). \end{array}$$

By differentiating both side with respect to time, we get

(9) $$\begin{array}{c} \frac{dN}{dt}=\frac{dS}{dt}+\frac{dV}{dt}+\frac{dV}{dt}+\frac{dR_{1}}{dt}+\frac{dR}{dt}+\frac{dR_{2}}{dt}+\frac{dI_{vr}}{dt}+\frac{dR_{3}}{dt},\\ \frac{dN}{dt}=\Lambda +\alpha R_{1}+\rho R_{2}+\theta R_{3}–\left(\lambda_{v}+\lambda_{r}+\mu \right)S+\lambda_{v}S–\left(\delta +\kappa \lambda_{r}+\mu \right)V+\delta V–\left(\varepsilon +\mu \right)U+\varepsilon U–\left(\alpha +\mu \right)R_{1}+\lambda_{r}S+\omega I_{vr}-\left(\sigma +\beta \lambda_{v}+\mu \right)+\sigma R-\left(\rho +\mu \right)R_{2}+\beta \lambda_{v}R+\kappa \lambda_{r}V-\left(\phi +\omega +\mu \right)I_{vr}+\phi I_{vr}-\left(\theta +\mu \right)R_{3},\\ \frac{dN}{dt}=\Lambda -\mu S-\mu V-\mu U-\mu R_{1}-\mu R-\mu R_{2}-\mu I_{vr}-\mu R_{3},\\ \frac{dN}{dt}=\Lambda -\mu \left(S+V+U+R_{1}+R+R_{2}+I_{vr}+R_{3}\right),\\ \frac{dN}{dt}\leq \Lambda -\mu \text{N}. \end{array}$$

Since all the state variables are nonnegative by Theorem 1, in the absence of infections, we have obtained (*dN*/*dt*) ≤ *Λ* − *μN*. By applying the standard comparison theorem, we have obtained ∫(*dN*/(*Λ* − *μN*)) ≤ ∫*dt*, and integrating both sides gives −(1/*μ*)ln(*Λ* − *μN*) ≤ *t* + *c*, where *c* is some constant. After some steps of calculations, we have obtained 0 ≤ *N* (*t*) ≤ (*Λ*/*μ*) which means all possible solutions of the system (3) with positive initial conditions enter in the bounded region (4).

## 3. Qualitative Analysis of the Model

### 3.1. Violence Submodel Analysis

In the absence of racism from the community of system (3), the model is said to be violence submodel which is obtained by making *R* = *I*_*vr*_ = *R*_2_ = *R*_3_ = 0 and *λ*_*v*_ = *β*_1_*V*; the violence submodel is

(10) $$\begin{array}{c} \frac{dS}{dt}=\Lambda +\alpha R_{1}–\left(\lambda_{v}+\mu \right)S,\\ \frac{dV}{dt}=\lambda_{v}S–\left(\delta +\mu \right)V,\\ \frac{dU}{dt}=\delta V–\left(\varepsilon +\mu \right)U,\\ \frac{dR_{1}}{dt}=\varepsilon U–\left(\alpha +\mu \right)R_{1}, \end{array}$$

with total population given by *N*_1_(*t*) = *S*(*t*) + *V*(*t*) + *U*(*t*) + *R*_1_(*t*).

#### 3.1.1. Violence-Free Equilibrium Point

In the absence of violence from the community, the timely independent solution of system (10) is said to be violence-free equilibrium point which is denoted by *E*_*v*_^0^ and obtained by making system (10) equal to zero with *V* = 0 is *E*_*v*_^0^ = (*S*_*v*_^0^, 0, 0, 0) = (*Λ*/*μ*, 0, 0, 0).

That is,

(11) $$\begin{array}{c} \frac{dS}{dt}=\Lambda +\alpha R_{1}–\left(\lambda_{v}+\mu \right)S=0,\\ \frac{dV}{dt}=\lambda_{v}S–\left(\delta +\mu \right)V=0,\\ \frac{dU}{dt}=\delta V–\left(\varepsilon +\mu \right)U=0,\\ \frac{dR_{1}}{dt}=\varepsilon U–\left(\alpha +\mu \right)R_{1}=0. \end{array}$$

Then, from *δV*–(*ε* + *μ*)*U* = 0, *U* = 0, from *εU*–(*α* + *μ*)*R*_1_ = 0, *R*_1_ = 0, *Λ* + *αR*_1_–(*λ*_*v*_ + *μ*)*S* = 0, *S* = *Λ*/*μ*.

Hence, *E*_*v*_^0^ = (*Λ*/*μ*, 0, 0, 0) is the violence-free equilibrium point of system (10).

#### 3.1.2. Basic Reproduction Number of Violence Submodel

In this submodel, we do have one infectious class *V* and use the method of next generation matrix to determine the basic reproduction number of violence submodel.

Take *X* = (*S*, *V*, *U*, *R*_1_)^*T*^ and system (10) rewritten as

(12) $$\begin{array}{c} \frac{dX}{dt}=f_{i}-v_{i}, \end{array}$$

where

(13) $$\begin{array}{c} f_{i}=\left(\begin{array}{c} \lambda_{v}S \end{array}\right)=\left(\beta_{1}SV\right),\\ f=\left(\begin{array}{c} \beta_{1}S^{0} \end{array}\right)=\left(\begin{array}{c} \frac{\beta_{1}\Lambda }{\mu } \end{array}\right),\\ v_{i}=\left(\begin{array}{c} \delta +\mu \end{array}\right)v,\\ v=\left(\begin{array}{c} \delta +\mu \end{array}\right),\\ v^{-1}=\frac{1}{\left(\delta +\mu \right)},\\ fv^{-1}=\frac{\beta_{1}\Lambda }{\mu \left(\delta +\mu \right)}. \end{array}$$

Thus, the spectral radius (the basic reproduction of violence infection submodel) of *fv*^−1^ is *ℜ*_0_^*v*^ = *β*_1_*Λ*/*μ*(*δ* + *μ*).

#### 3.1.3. Violence-Persistence Equilibrium Point

In the presence of violence in the population, the time dependent solution of the system (10) is said to be violence-persistence equilibrium point denoted by *E*_*v*_^∗^ and defined as *E*_*v*_^∗^ = (*S*_*v*_^∗^, *U*_*v*_^∗^, *V*_*v*_^∗^, *R*_1*v*_^∗^), and after some steps of calculations, we have obtained

(14) $$\begin{array}{c} S_{v}^{*}=\frac{\Lambda \left(\alpha +\mu \right)\left(\varepsilon +\mu \right)\left(\delta +\mu \right)}{\left(\left(\alpha +\mu \right)\left(\lambda_{v}^{*}+\mu \right)\left(\varepsilon +\mu \right)\left(\delta +\mu \right)-\alpha \varepsilon \delta \lambda_{v}^{*}\right)},\\ U_{v}^{*}=\frac{\Lambda \delta \lambda_{v}^{*}\left(\alpha +\mu \right)}{\left(\left(\alpha +\mu \right)\left(\lambda_{v}^{*}+\mu \right)\left(\varepsilon +\mu \right)\left(\delta +\mu \right)-\alpha \varepsilon \delta \lambda_{v}^{*}\right)},\\ V_{v}^{*}=\frac{\Lambda \lambda_{v}^{*}\left(\alpha +\mu \right)\left(\varepsilon +\mu \right)}{\left(\left(\alpha +\mu \right)\left(\lambda_{v}^{*}+\mu \right)\left(\varepsilon +\mu \right)\left(\delta +\mu \right)-\alpha \varepsilon \delta \lambda_{v}^{*}\right)},\\ R_{1v}^{*}=\frac{\Lambda \delta \varepsilon \lambda_{v}^{*}}{\left(\left(\alpha +\mu \right)\left(\lambda_{v}^{*}+\mu \right)\left(\varepsilon +\mu \right)\left(\delta +\mu \right)-\alpha \varepsilon \delta \lambda_{v}^{*}\right)}. \end{array}$$

**Theorem 3 .**

Violence-persistence equilibrium point of system (10) is unique if and only if *ℜ*_0_^*v*^ > 1.

**Proof**

Using violence force of infection, we have

(15) $$\begin{array}{c} \lambda_{v}^{*}=\beta_{1}V^{*}=\frac{\beta_{1}\Lambda \lambda_{v}^{*}\left(\alpha +\mu \right)\left(\varepsilon +\mu \right)}{\left(\left(\alpha +\mu \right)\left(\lambda_{v}^{*}+\mu \right)\left(\varepsilon +\mu \right)\left(\delta +\mu \right)-\alpha \varepsilon \delta \lambda_{v}^{*}\right)}. \end{array}$$

The nonzero value of *λ*_*v*_^∗^ from equation (15) is

(16) $$\begin{array}{c} \lambda_{v}^{*}=\frac{\left(\alpha +\mu \right)\left(\varepsilon +\mu \right)\mu \left(\delta +\mu \right)\left(\left(\beta_{1}\Lambda /\mu \left(\delta +\mu \right)\right)-1\right)}{\left(\left(\alpha +\mu \right)\left(\varepsilon +\mu \right)\left(\delta +\mu \right)-\alpha \varepsilon \delta \right)}=\frac{\left(\alpha +\mu \right)\left(\varepsilon +\mu \right)\mu \left(\delta +\mu \right)\left(R_{0}^{v}-1\right)}{\left(\left(\alpha +\mu \right)\left(\varepsilon +\mu \right)\left(\delta +\mu \right)-\alpha \varepsilon \delta \right)}>0\text{ if and only if }R_{0}^{v}>1. \end{array}$$

Hence, violence submodel has unique violence-persistence equilibrium point iff *ℜ*_0_^*v*^ > 1.

**Theorem 4 .**

The violence-free equilibrium point of system (10) is locally asymptotically stable if *ℜ*_0_^*v*^ < 1, otherwise unstable.

**Proof**

The Jacobian matrix of system (10) at the violence-free equilibrium point is

(17) $$\begin{array}{c} J\left(E_{v}^{0}\right)=\left(\begin{array}{cccc} –\mu & \frac{–\beta_{1}\Lambda }{\mu } & 0 & \alpha \\ 0 & \;\frac{\beta_{1}\Lambda -\mu \left(\delta +\mu \right)}{\mu } & 0 & 0\\ 0 & \delta & –\left(\varepsilon +\mu \right) & 0\\ 0 & 0 & \varepsilon & –\left(\alpha +\mu \right) \end{array}\right). \end{array}$$

From the Jacobian matrix, the characteristic equation is

(18) $$\begin{array}{c} \begin{array}{c} \left|\begin{array}{cccc} –\mu -\lambda & \frac{–\beta_{1}\Lambda }{\mu } & 0 & \alpha \\ 0 & \frac{\beta_{1}\Lambda -\mu \left(\delta +\mu \right)}{\mu }-\lambda & 0 & 0\\ 0 & \delta & –\left(\varepsilon +\mu \right)-\lambda & 0\\ 0 & 0 & \varepsilon & –\left(\alpha +\mu \right)-\lambda \end{array}\right|=0,\\ \left(–\mu -\lambda \right)\left(\frac{\beta_{1}\Lambda -\mu \left(\delta +\mu \right)}{\mu }-\lambda \right)\left(–\left(\varepsilon +\mu \right)-\lambda \right)\left(–\left(\alpha +\mu \right)-\lambda \right)=0, \end{array} \end{array}$$

which gives the corresponding eigenvalues

(19) $$\begin{array}{c} \lambda_{1}=–\mu <0,\\ \lambda_{2}=–\left(\varepsilon +\mu \right)<0,\\ \lambda_{3}=–\left(\alpha +\mu \right)<0,\\ \lambda_{4}=\left(\delta +\mu \right)\left(R_{0}^{v}-1\right)<0. \end{array}$$

Those all eigenvalues are negative which implies that the violence-free equilibrium point of violence submodel is locally asymptotically stable if  *ℜ*_0_^*v*^ < 1.

**Theorem 5 .**

The violence-free equilibrium point of system (10) is globally asymptotically stable if  *ℜ*_0_^*v*^ < 1, otherwise unstable.

**Proof**

Consider the Lyapunov function *l*(*V*) = *aV*, where *a* = 1/(*δ* + *μ*), therefore,

(20) $$\begin{array}{c} l\left(V\right)=\frac{1}{\left(\delta +\mu \right)}V,\\ \frac{dl}{dt}=\frac{1}{\left(\delta +\mu \right)}\frac{d\text{V}}{dt},\\ \frac{dl}{dt}=\frac{1}{\left(\delta +\mu \right)}\left(\lambda_{v}S–\left(\delta +\mu \right)\right.V,\\ \frac{dl}{dt}\leq \frac{1}{\left(\delta +\mu \right)}\left(\lambda_{v}S_{v}^{0}–\left(\delta +\mu \right)\right)V,\\ \frac{dl}{dt}\leq \frac{\mu \left(\delta +\mu \right)}{\left(\delta +\mu \right)}\left(\frac{\left(\beta_{1}\Lambda /\mu \left(\delta +\mu \right)\right)-1}{\mu }\right)V,\\ \frac{dl}{dt}\leq \left(\;R_{0}^{v}-1\right)V,\\ \frac{dl}{dt}<0\text{ if and only if }R_{0}^{v}<1. \end{array}$$

Thus, violence-free equilibrium of system (10) is globally asymptotically stable when  *ℜ*_0_^*v*^ < 1.

### 3.2. Racism Submodel Analysis

In the absence of violence from the community of system (3), the model is said to be racism submodel which is obtained by making *V* = *U* = *I*_*vr*_ = *R*_1_ = *R*_3_ = 0 and *λ*_*r*_ = *β*_2_*R*.

The racism submodel is

(21) $$\begin{array}{c} \frac{dS}{dt}=\Lambda +\rho R_{2}–\left(\lambda_{r}+\mu \right)S,\\ \frac{dR}{dt}=\lambda_{r}S-\left(\sigma +\mu \right)R,\\ \frac{dR_{2}}{dt}=\sigma R-\left(\rho +\mu \right)R_{2}, \end{array}$$

with total population given by *N*_2_(*t*) = *S*(*t*) + *R*(*t*) + *R*_2_(*t*).

#### 3.2.1. Racism-Free Equilibrium Point

In the absence of racism from the community, the timely independent solution of system (21) is said to be racism-free equilibrium point which is denoted by *E*_*r*_^0^ and obtained by making system (21) equals to zero with *R* = 0 is *E*_*r*_^0^ = (*S*_*r*_^0^, 0, 0) = (*Λ*/*μ*, 0, 0).

That is,

(22) $$\begin{array}{c} \frac{dS}{dt}=\Lambda +\rho R_{2}–\left(\lambda_{r}+\mu \right)S=0,\\ \frac{dR}{dt}=\lambda_{r}S-\left(\sigma +\mu \right)R=0,\\ \frac{dR_{2}}{dt}=\sigma R-\left(\rho +\mu \right)R_{2}=0. \end{array}$$

Then, from *σR* − (*ρ* + *μ*)*R*_2_ = 0, *R*_2_ = 0, and from *Λ* + *ρR*_2_–(*λ*_*r*_ + *μ*)*S* = 0, *S* = *Λ*/*μ*.

Hence, *E*_*r*_^0^ = (*Λ*/*μ*, 0, 0) is the racism-free equilibrium point of system (21).

#### 3.2.2. Racism Submodel Basic Reproduction Number

In this submodel, we do have one infectious class *R* and use the method of next generation matrix approach to determine the basic reproduction number of racism submodel.

Take *X* = (*S*, *R*, *R*_2_)^*T*^, and system (21) can be rewritten as

(23) $$\begin{array}{c} \frac{dX}{dt}=f_{i}-v_{i}, \end{array}$$

where

(24) $$\begin{array}{c} f_{i}=\left(\begin{array}{c} \lambda_{r}S \end{array}\right)=\left(\beta_{2}SR\right),\\ f=\left(\begin{array}{c} \beta_{1}S_{r}^{0} \end{array}\right)=\left(\begin{array}{c} \frac{\beta_{2}\Lambda }{\mu } \end{array}\right),\\ v_{i}=\left(\sigma +\mu \right)R,\\ v=\left(\sigma +\mu \right),\\ v^{-1}=\frac{1}{\left(\sigma +\mu \right)},\\ fv^{-1}=\frac{\beta_{2}\Lambda }{\mu \left(\sigma +\mu \right)}. \end{array}$$

Thus, the spectral radius (the basic reproduction of violence infection submodel) of *fv*^−1^ is *ℜ*_0_^*r*^ = *β*_2_*Λ*/*μ*(*σ* + *μ*).

#### 3.2.3. Racism-Persistence Equilibrium Point of Racism Submodel

In the presence of racism under the population, the timely dependent solution of the system (21) is said to be racism-persistence equilibrium point denoted by *E*_*r*_^∗^ and given by *E*_*r*_^∗^ = (*S*_*r*_^∗^, *R*_*r*_^∗^, *R*_2*r*_^∗^), and after some steps of calculations, we have obtained

(25) $$\begin{array}{c} S_{r}^{*}=\frac{\Lambda \left(\rho +\mu \right)\left(\sigma +\mu \right)}{\left(\rho +\mu \right)\left(\sigma +\mu \right)\left(\lambda_{r}^{*}+\mu \right)-{\rho \sigma \lambda }_{r}^{*}},\\ R_{r}^{*}=\frac{\Lambda \left(\rho +\mu \right)\left(\sigma +\mu \right)\lambda_{r}^{*}}{\left(\rho +\mu \right){\left(\sigma +\mu \right)}^{2}\left(\lambda_{r}^{*}+\mu \right)-\left(\sigma +\mu \right){\rho \sigma \lambda }_{r}^{*}},\\ R_{2r}^{*}=\frac{\sigma \Lambda \left(\rho +\mu \right)\left(\sigma +\mu \right)\lambda_{r}^{*}}{{\left(\rho +\mu \right)}^{2}{\left(\sigma +\mu \right)}^{2}\left(\lambda_{r}^{*}+\mu \right)-\left(\rho +\mu \right)\left(\sigma +\mu \right){\rho \sigma \lambda }_{r}^{*}}. \end{array}$$

**Theorem 6 .**

Racism-persistence equilibrium point of system (21) is unique if and only if *ℜ*_0_^*r*^ > 1.

**Proof**

The racism force of infection is *λ*_*r*_ = *β*_2_*R*.

Then, substitute *R*_*r*_^∗^ in *λ*_*r*_ = *β*_2_*R* as

(26) $$\begin{array}{c} \lambda_{r}^{*}=\beta_{2}R_{r}^{*}=\frac{\beta_{2}\Lambda \left(\rho +\mu \right)\left(\sigma +\mu \right)\lambda_{r}^{*}}{\left(\rho +\mu \right){\left(\sigma +\mu \right)}^{2}\left(\lambda_{r}^{*}+\mu \right)-\left(\sigma +\mu \right){\rho \sigma \lambda }_{r}^{*}}. \end{array}$$

The nonzero solution of equation (26) is *λ*_*r*_^∗^ = ((*ρ* + *μ*)*μ*(*σ* + *μ*)(*ℜ*_0_^*r*^ − 1)/((*ρ* + *μ*)(*σ* + *μ*) − *ρσ*)) > 0 if and only if *ℜ*_0_^*r*^ > 1.

Hence, the system (21) has unique racism-persistence equilibrium point if and only if *ℜ*_0_^*r*^ > 1.

**Theorem 7 .**

The racism-free equilibrium point of system (21) is locally asymptotically stable if *ℜ*_0_^*r*^ < 1, otherwise unstable

**Proof**

The Jacobian matrix of system (21) at racism-free equilibrium point is

(27) $$\begin{array}{c} J\left(E_{r}^{*}\right)=\left(\begin{array}{ccc} –\mu & \frac{–\beta_{2}\Lambda }{\mu } & 0\\ \frac{\beta_{2}\Lambda }{\mu } & \frac{\beta_{2}\Lambda -\mu \left(\sigma +\mu \right)}{\mu } & 0\\ 0 & \sigma & –\left(\rho +\mu \right) \end{array}\right). \end{array}$$

The characteristic equation of *J*(*E*_*r*_^0^) is

(28) $$\begin{array}{c} \left|\begin{array}{ccc} –\mu -\lambda & \frac{–\beta_{2}\Lambda }{\mu } & 0\\ \frac{\beta_{2}\Lambda }{\mu } & \frac{\beta_{2}\Lambda -\mu \left(\sigma +\mu \right)}{\mu }-\lambda & 0\\ 0 & \sigma & –\left(\rho +\mu \right)-\lambda \end{array}\right|=0,\\ \left(–\mu -\lambda \right)\left(\frac{\beta_{2}\Lambda -\mu \left(\sigma +\mu \right)}{\mu }-\lambda \right)\left(–\left(\rho +\mu \right)-\lambda \right)+\frac{\beta_{2}\Lambda }{\mu }*\frac{\beta_{2}\Lambda }{\mu }\left(–\left(\rho +\mu \right)-\lambda \right)=0,\\ \lambda_{1}=–\left(\rho +\mu \right),\text{or }\left(–\mu -\lambda \right)\left(\frac{\beta_{2}\Lambda -\mu \left(\sigma +\mu \right)}{\mu }-\lambda \right)+\frac{\beta_{2}\Lambda }{\mu }*\frac{\beta_{2}\Lambda }{\mu }=0,\\ \lambda^{2}+\left(\mu -\left(\sigma +\mu \right)\left(R_{0}^{r}-1\right)\right)\lambda +\mu \left(\sigma +\mu \right)\left(1-R_{0}^{r}\right)+\frac{\beta_{2}\Lambda }{\mu }\frac{\beta_{2}\Lambda }{\mu }=0. \end{array}$$

It can be written as *a*_0_*λ*^2^ + *a*_1_*λ* + *a*_2_ = 0, where

(29) $$\begin{array}{c} a_{0}=1,\\ a_{1}=\left(\mu -\left(\sigma +\mu \right)\left(R_{0}^{r}-1\right)\right)>0,\text{iff }R_{0}^{r}<1,\\ a_{2}=\mu \left(\sigma +\mu \right)\left(1-R_{0}^{r}\right)+\frac{\beta_{2}\Lambda }{\mu }*\frac{\beta_{2}\Lambda }{\mu }>0,\text{iff }R_{0}^{r}<1. \end{array}$$

Hence, all eigenvalues are negative if and only if *ℜ*_0_^*r*^ < 1. Thus, racism-free equilibrium point is locally asymptotically stable if *ℜ*_0_^*r*^ < 1.

**Theorem 8 .**

The racism-free equilibrium point of system (21) is globally asymptotically stable if *ℜ*_0_^*r*^ < 1, otherwise unstable.

**Proof**

Consider the Lyapunov function *l*(*R* ) = *aR*, where *a* = 1/(*σ* + *μ*)

(30) $$\begin{array}{c} l\left(R\;\right)=\frac{R}{\left(\sigma +\mu \right)},\\ \frac{dl}{dt}=\frac{1}{\left(\sigma +\mu \right)}\left(\lambda_{r}S-\left(\sigma +\mu \right)R\right),\\ \frac{dl}{dt}=\frac{1}{\left(\sigma +\mu \right)}\left(\beta_{2}S-\left(\sigma +\mu \right)\right)R,\\ \frac{dl}{dt}\leq \frac{1}{\left(\sigma +\mu \right)}\left(\beta_{2}S^{0}-\left(\sigma +\mu \right)\right)R,\\ \frac{dl}{dt}\leq \frac{1}{\left(\sigma +\mu \right)}\left(\frac{\beta_{2}\Lambda }{\mu }-\left(\sigma +\mu \right)\right)R,\\ \frac{dl}{dt}\leq \frac{1}{\left(\sigma +\mu \right)}\left(\frac{\beta_{2}\Lambda -\mu \left(\sigma +\mu \right)}{\mu }\right)R,\\ \frac{dl}{dt}\leq \frac{\mu \left(\sigma +\mu \right)}{\left(\sigma +\mu \right)}\left(\frac{\left(\beta_{2}\Lambda /\mu \left(\sigma +\mu \right)\right)-1}{\mu }\right)R,\\ \frac{d\text{l}}{dt}\leq \frac{\mu \left(\sigma +\mu \right)}{\mu \left(\sigma +\mu \right)}\left(R_{0}^{r}-1\right)R,\\ \frac{d\text{l}}{dt}<0,\text{if }{R_{0}}^{r}<1. \end{array}$$

Thus, the racism-free equilibrium point is globally asymptotically stable if *ℜ*_0_^*r*^ < 1.

### 3.3. Violence and Racism Coexistence Full Model Analysis

#### 3.3.1. Coexistence Free Equilibrium Point

The coexistence free equilibrium point of the full model is obtained by making system (3) equal to zero with *V* = *U* = *R* = *R*_1_ = *R*_2_ = *R*_3_ = 0, and it is given by

(31) $$\begin{array}{c} E_{vr}^{0}=\left(S^{0},V^{0},U^{0},R^{0},I_{vr}^{0},R_{1}^{0},R_{2}^{0},R_{3}^{0}\right)=\left(\frac{\Lambda }{\mu },0,0,0,0,0,0,0\right). \end{array}$$

#### 3.3.2. Basic Reproduction Number of the Full Model

In this study, we compute the violence-racism coexistence model basic reproduction number denoted by  *ℛ*_0_^*vr*^ using next-generation matrix criteria by Van den Driessche and Watmough [39]. In this model, we do have three infectious classes; those are *V*, *R*, and *I*_*vr*_; then, we have

(32) $$\begin{array}{c} f_{i}=\left(\begin{array}{c} \lambda_{v}S\\ \lambda_{r}S\\ \beta \lambda_{v}R+\kappa \lambda_{r}V \end{array}\right)=\left(\begin{array}{c} \beta_{1}\left(V+\theta_{2}I_{vr}\right)S\\ \beta_{2}\left(R+\theta_{1}I_{vr}\right)S\\ \beta_{1}\beta \left(V+\theta_{2}I_{vr}\right)R+\beta_{2}\kappa \left(R+\theta_{1}I_{vr}\right)V \end{array}\right),\\ f=\left(\begin{array}{ccc} \beta_{1}S^{0} & 0 & \beta_{1}\theta_{2}S^{0}\\ 0 & \beta_{2}S^{0} & \beta_{2}\theta_{1}S^{0}\\ 0 & 0 & 0 \end{array}\right)=\left(\begin{array}{ccc} \frac{\beta_{1}\Lambda }{\mu } & 0 & \frac{\beta_{1}\theta_{2}\Lambda }{\mu }\\ 0 & \frac{\beta_{2}\Lambda }{\mu } & \frac{\beta_{2}\theta_{1}\Lambda }{\mu }\\ 0 & 0 & 0 \end{array}\right),\\ v_{i}={v_{i}}^{-}\left(x\right)-{v_{i}}^{+}\left(x\right)=\left(\begin{array}{c} \left(\delta +\kappa \lambda_{r}+\mu \right)V\\ \left(\sigma +\beta \lambda_{v}+\mu \right)R\\ -\left(\phi +\omega +\mu \right)I_{vr} \end{array}\right),\\ v=\left(\begin{array}{ccc} \left(\delta +\mu \right) & 0 & 0\\ 0 & \left(\sigma +\mu \right) & 0\\ 0 & 0 & \left(\phi +\omega +\mu \right) \end{array}\right),\\ v^{-1}=\left(\begin{array}{ccc} \frac{1}{\left(\delta +\mu \right.} & 0 & 0\\ 0 & \frac{1}{\sigma +\mu } & 0\\ 0 & 0 & \frac{1}{\phi +\omega +\mu } \end{array}\right),\\ {fv}^{-1}=\left(\begin{array}{ccc} \frac{\beta_{1}\Lambda }{\mu \left(\delta +\mu \right)} & \frac{\beta_{1}\Lambda }{\mu \left(\sigma +\mu \right)} & \frac{\beta_{1}\theta_{2}\Lambda }{\mu \left(\phi +\omega +\mu \right)}\\ 0 & \frac{\beta_{2}\Lambda }{\mu \left(\sigma +\mu \right)} & \frac{\beta_{2}\theta_{1}\Lambda }{\mu \left(\phi +\omega +\mu \right)}\\ 0 & 0 & 0 \end{array}\right). \end{array}$$

The nonzero eigenvalues of *fv*^−1^ are *λ*_1_ = *β*_1_*Λ*/*μ*(*δ* + *μ*), or *λ*_2_ = *β*_2_*Λ*/*μ*(*σ* + *μ*).

Hence, the basic reproduction number of full model (3) is

*ℜ*_0_^*vr*^ = max{*λ*_1_, *λ*_2_} = max{*ℜ*_0_^*v*^, *ℜ*_0_^*r*^}, where *ℜ*_0_^*v*^ = *β*_1_*Λ*/*μ*(*δ* + *μ*) and *ℜ*_0_^*r*^ = *β*_2_*Λ*/*μ*(*σ* + *μ*).

#### 3.3.3. Coexistence Free Equilibrium Point Local Stability

**Theorem 9 .**

The coexistence free equilibrium point of a full model is locally asymptotically stable if *ℜ*_0_^*vr*^ < 1, otherwise unstable.

**Proof**

The Jacobian matrix of the full coexistence model is

(33) $$\begin{array}{c} J\left(E^{o}\right)=\left(\begin{array}{cccccccc} -\mu & -\beta_{1}S^{0} & 0 & \alpha & -\beta_{2}S^{0} & \rho & D_{3} & \theta \\ 0 & D_{1} & 0 & 0 & 0 & 0 & \beta_{1}\theta_{2}S^{0} & 0\\ 0 & \delta & –\left(\varepsilon +\mu \right) & 0 & 0 & 0 & 0 & 0\\ 0 & 0 & \varepsilon & –\left(\alpha +\mu \right) & 0 & 0 & 0 & 0\\ 0 & 0 & 0 & 0 & D_{2} & 0 & D_{4} & 0\\ 0 & 0 & 0 & 0 & \sigma & -\left(\rho +\mu \right) & 0 & 0\\ 0 & 0 & 0 & 0 & 0 & 0 & -\left(\phi +\omega +\mu \right) & 0\\ 0 & 0 & 0 & 0 & 0 & 0 & \phi & -\left(\theta +\mu \right) \end{array}\right), \end{array}$$

where *D*_1_ = *β*_1_*S*^0^ − (*δ* + *μ*), *D*_2_ = *β*_2_*S*^0^ − (*δ* + *μ*), *D*_3_ = −(*β*_1_*θ*_2_ + *β*_2_*θ*_1_)*S*^0^, *D*_4_ = *β*_2_*θ*_1_*S*^0^ + *ω*, and *D*_5_ = −(*ϕ* + *ω* + *μ*).

The characteristic equation of the Jacobian matrix *J*(*E*^*o*^) is

(34) $$\begin{array}{c} \left|\begin{array}{cccccccc} -\mu -\lambda & -\beta_{1}S^{0} & 0 & \alpha & -\beta_{2}S^{0} & \rho & D_{3} & \theta \\ 0 & D_{1} & 0 & 0 & 0 & 0 & \beta_{1}\theta_{2}S^{0} & 0\\ 0 & \delta & –\left(\varepsilon +\mu \right)-\lambda & 0 & 0 & 0 & 0 & 0\\ 0 & 0 & \varepsilon & –\left(\alpha +\mu \right)-\lambda & 0 & 0 & 0 & 0\\ 0 & 0 & 0 & 0 & D_{2} & 0 & D_{4} & 0\\ 0 & 0 & 0 & 0 & \sigma & -\left(\rho +\mu \right)-\lambda & 0 & 0\\ 0 & 0 & 0 & 0 & 0 & 0 & -\lambda -{\text{D}}_{5} & 0\\ 0 & 0 & 0 & 0 & 0 & 0 & \phi & -\left(\theta +\mu \right)-\lambda \end{array}\right|=0,\\ \left(-\mu -\lambda \right)\left(\beta_{1}S^{0}-\left(\delta +\mu \right)-\lambda \right)\left(–\left(\varepsilon +\mu \right)-\lambda \right)\left(–\left(\alpha +\mu \right)-\lambda \right)\left(\beta_{2}S^{0}-\left(\delta +\mu \right)-\lambda \right)\left(-\left(\rho +\mu \right)-\lambda \right)\left(-\left(\phi +\omega +\mu \right)-\lambda \right)\left(-\left(\theta +\mu \right)-\lambda \right)=0. \end{array}$$

Then, after some simplification, we have obtained

(35) $$\begin{array}{c} \lambda_{1}=-\mu <0,\lambda_{2}=\left(\delta +\mu \right)\left(R_{0}^{v}-1\right)<0\text{ if }R_{0}^{v}<1,\lambda_{3}=–\left(\varepsilon +\mu \right)<0,\lambda_{4}=–\left(\alpha +\mu \right)<0,\lambda_{5}=\left(\delta +\mu \right)\left(R_{0}^{r}-1\right)\text{ if }R_{0}^{r}<1,\lambda_{6}=-\left(\rho +\mu \right)<0,\lambda_{7}=-\left(\phi +\omega +\mu \right)<0,\lambda_{8}=-\left(\theta +\mu \right)<0. \end{array}$$

Hence, the coexistence free equilibrium point of system (3) is locally asymptotically stable whenever *ℜ*_0_^*vr*^ < 1.

## 4. Sensitivity Analysis and Numerical Simulations

In this section, we convey both the sensitivity analysis and numerical simulations to verify the qualitative results of our mathematical model (3). Particularly, some numerical verification is considered to illustrate the qualitative analysis and results of the preceding sections. Here, we have taken some parameter values from literatures and assume some of the parameter values that are not from real data, since there is the lack of mathematical model analysis literatures which have been done to study the dynamics of violence-racism coexistence in the community.

### 4.1. Sensitivity Analysis

**Definition 1 .**

The normalized forward sensitivity index of a variable violence-racism coexistence reproduction number *ℜ*_0_^*vr*^ for the coexistence model (3) that depends differentially on a parameter *ζ* is defined as SI(*p*) = *∂ℜ*_0_^*vr*^/*∂ζ*∗*ζ*/*ℜ*_0_^*vr*^ [27, 28].

The violence-racism coexistence sensitivity indices allow us to justify the relative importance of various parameters in the violence-racism coexistence incidence and prevalence. The most sensitive parameter has the magnitude of the sensitivity index greater than all other parameters. In this study, we computed the sensitivity index in terms of *ℜ*_0_^*vr*^.

Taking the values of parameters given in Table 2, the sensitivity indices are calculated in Table 3 and Table 4 as

In the study, with the given parameter values in Table 2, we have computed *ℜ*_0_^*v*^ = 3.7 at the violence spreading rate *β*_1_ = 0.003 which imply that violence spreads throughout the community. Also, we have obtained the sensitivity indices given in Table 3. Moreover, sensitivity analysis given in Table 3 explains that the human population recruitment rate *Λ* and violence transmission rate *β*_1_ are highly affecting the violence reproduction number *ℜ*_0_^*v*^.

Moreover, with the given parameter values in Table 2, we have computed *ℜ*_0_^*r*^ = 6.9 at the racism spreading rate *β*_2_ = 0.007 which imply that racism spreads throughout the community; also, we have obtained the sensitivity indices given in Table 4. Moreover, sensitivity analysis given in Table 4 explains that the human population recruitment rate *Λ* and racism transmission rate *β*_2_ are highly affecting the racism reproduction number *ℜ*_0_^*r*^.

### 4.2. Numerical Simulations

#### 4.2.1. Simulations of the Model Thresholds

Using Table 2 data, we have obtained *ℜ*_0_^*vr*^ = max{*ℜ*_0_^*v*^, *ℜ*_0_^*r*^} = max{3.7, 6.9} = 6.9 > 1, and from the sensitivity indices calculation results of Table 4, we can identify some parameters that strongly influence the violence-racism coexistence model dynamics. Parameter  *β*_2_ has a positive impact on the basic reproduction number *ℜ*_0_^*vr*^; that is, an increase in  *β*_2_ implies an increase in *ℜ*_0_^*vr*^ = *ℜ*_0_^*r*^. Similarly, parameter *σ* has a negative impact on the basic reproduction number *ℜ*_0_^*vr*^; that is, an increase in the value of *σ* implies a decrement in *ℜ*_0_^*vr*^ = *ℜ*_0_^*r*^.

Figure 2 illustrates that whenever the value of the racism transmission rate increases, the coexistence reproduction number *ℜ*_0_^*vr*^ = *ℜ*_0_^*r*^ highly increases.

Figure 3 illustrates that whenever the value of the racism recovery rate increases, then the coexistence reproduction number *ℜ*_0_^*vr*^ = *ℜ*_0_^*r*^ decreases.

#### 4.2.2. Simulations for the Full Dynamical System

Figure 4 shows us the trajectory simulation of the violence-racism coexistence model with parameter values given in Table 2 and *β*_2_ = 0.0002, where the violence-racism coexistence model basic reproduction number is *ℜ*_0_^*vr*^ = *ℜ*_0_^*r*^ = 0.32. Meaning, in the long run (after 10 years), we can see that the violence-racism coexistence state eradicates in the community. That means that the solutions of the model converge to the violence-racism coexistence free equilibrium point.

Figure 5 shows us the trajectory simulation of the violence-racism coexistence model with parameter values given in Table 2 and *β*_2_ = 0.004, where the violence-racism coexistence model basic reproduction number is *ℜ*_0_^*vr*^ = *ℜ*_0_^*r*^ = 6.9. Meaning, in the long run (after 12 years), we can see that the violence-racism coexistence state persists in the community and stabilizes in time. That means the solutions of the model converge to the violence-racism coexistence endemic equilibrium point. Furthermore, the simulation shows that the less recovery rate of the violence-racism coinfectious individuals leads to the prevalence of violence-racism coexistence spread.

#### 4.2.3. Simulations of Coinfectious Variable

Figure 6 illustrates the impact of violence only controlling rate *ω* on violence-racism coinfectious individuals *I*_*vr*_, which means we set the impact of the rate *ω* as we increase values 0.6, 0.7, and 0.8. In Figure 6, we can see that the number of violence-racism coinfectious individuals decreases as *ω* increases. Similarly, Figure 7 illustrates us that the result of violence-racism coinfectious individuals decreases whenever the controlling rate *ϕ* increases from 0.6 to 0.8.

## 5. Discussions and Conclusions

In this newly proposed social science discipline mathematical model study, we have constructed and analyzed the first and new compartmental mathematical model on violence and racism coexistence behaviors in a community with the attempting of applying possible control measures. Like infectious diseases, in this study, we have interchangeably applied persistence and coexistence as infection and coinfection, respectively. We have determined and shown the positivity and boundedness of the model solutions in a mathematically and physically meaningfully feasible region. The equilibrium points and the basic reproduction numbers are determined by using next generator operator method. In addition, we analyzed the local and global stability of all equilibria.

Using sensitivity analysis and numerical simulations, we have verified the detailed theoretical results such that applying data given in Table 2, the basic reproduction number of the coinfection is the maximum of the two submodel reproduction numbers given by *ℜ*_0_^*vr*^ = max{*ℜ*_0_^*v*^, *ℜ*_0_^*r*^} = max{3.7, 6.9} = *ℜ*_0_^*r*^ = 6.9 > 1 at *β*_1_ = 0.003 and *β*_2_ = 0.007 which implies that the coinfection is spreading through the considered community. Sensitivity analysis shows that transmission rates are the most positively influencing parameters. On the other hands, the recuperated rate *σ* and the negotiated rate *δ* are the most negatively influencing parameters.

Figure 2 reflects that increasing the value of the racism transmission rate increases the basic reproduction number *ℜ*_0_^*vr*^ = *ℜ*_0_^*r*^ of the coinfectious population. Figure 3 reflects that whenever we increase the value of the racism recovery rate by applying the general controlling strategies, the coexistence reproduction number *ℜ*_0_^*vr*^ = *ℜ*_0_^*r*^ decreases. Figure 4 shows the trajectory of the violence-racism coexistence model with given constant parameter values at *β*_1_ = 0.0001 and *β*_2_ = 0.0002, and the basic reproduction number is *ℜ*_0_^*vr*^ = 0.32. It implies that in the long run (after 10 years), the violence-racism coexistence state eradicates from the community. That means that the solutions of the model converge to the violence-racism coexistence free equilibrium point. Figure 5 shows the trajectory simulation of the violence-racism coexistence model with given constant parameter values at *β*_1_ = 0.001 and *β*_2_ = 0.004; the violence-racism coexistence model basic reproduction number is *ℜ*_0_^*vr*^ = *ℜ*_0_^*r*^ = 6.9; it means, in the long run (after 20 years), the violence-racism coexistence state persists in the community and stabilizes in time. That means that the solutions of the model converge to the violence-racism coexistence prevalence equilibrium point.

Figures 6 and 7 illustrate the impact of violence only controlling rate *ω* and violence-racism coinfection general controlling rate *ϕ* on violence-racism coinfectious individuals *I*_*vr*_, which means if we increase the values of *ω* and *ϕ* from 0.6 to 0.8, the violence-racism coinfectious individuals decreases. Finally, we recommend for both the social sciences experts and the public health stakeholders to decrease the spreading rates and to maximize the general controlling mechanisms (negotiated and recovery rates) of the violence-racism coinfectious individuals.

Finally, we recommend for the governments of nations to introduce, apply, and ensure antiracism and antiviolence laws and take the bold measures to break the interconnection of violence and racism. We want to remark the whole community to stay united to identify common problems and committed to research and advocacy from societies. The international institutions shall be collaborated for better understanding of these two interlinked problems and set up monitoring and investigation bodies. The limitations of this study are as follows: the next potential researchers can incorporate and extend them; this study will be optimal control approach, stochastic approach, fractional order derivative approach, environmental impacts, and age and spatial structures, whenever possible validate the model by applying appropriate real data.

## Figures and Tables

**Figure 1:** The flow diagram of violence and racism coexistence transmission dynamics.

**Figure 2:** *ℜ*_0_^*vr*^ = *ℜ*_0_^*r*^ versus the transmission rate *β*2.

**Figure 3:** *ℜ*_0_^*vr*^ = *ℜ*_0_^*r*^ versus the recovery rate *σ*.

**Figure 4:** Behaviors of the model solutions whenever *ℜ*_0_^*vr*^ = *ℜ*_0_^*r*^ < 1.

**Figure 5:** Behaviors of the model solutions whenever *ℜ*_0_^*vr*^ = *ℜ*_0_^*r*^ > 1.

**Figure 6:** Effect of *ω* on coinfectious individuals *I*_*vr*_.

**Figure 7:** Effect of *ϕ* on coinfectious individuals *I*_*vr*_.

**Table 1:** Description of biological parameters.

Parameter	Biological description
*Λ*	Recruitment rate of susceptible individuals
*β*	The modification parameter
*β*_1_	Violence transmission rate
*β*_2_	Racism transmission rate
*δ*	The negotiated rate of violated individuals
*ε*	The recuperated rate of negotiated individuals
*α*	The conversion rate of recuperated individual to susceptible
*ω*	The controlling rate of violence from violence and racism coexistence class
*κ*	The modification parameter
*σ*	The recuperated rate of racist individuals
*ρ*	The rate of individuals those who stopped racism purely
*ϕ*	Recuperated rate of violence-racism coexistence
*θ*	The rate of individuals those who stopped both violence and racism purely
*μ*	Individual's natural death rate

**Table 2:** Parameter values for numerical simulation.

Parameter	Value	Source
*μ*	0.01	[8, 9]
*Λ*	50	[1, 9]
*α*	0.51	Assume
*ε*	0.60	Assume
*σ*	0.50	Assume
*δ*	0.40	Assume
*κ*	1.3	Assume
*ρ*	0.61	Assume
*θ*	0.72	Assume
*β*	1.2	Assume
*β*_1_	Variable	Assume
*β*_2_	Variable	Assume
*ω*	0.60	Assume
*ϕ*	0.50	Assume
*ω*	0.42	Assume

**Table 3:** Sensitivity indices of *ℜ*_0_^*v*^.

Sensitivity index	Sensitivity indices
SI(*β*_1_)	+1
SI(*Λ*)	+1
SI(*δ*)	-0.81
SI(*μ*)	-0.31

**Table 4:** Sensitivity indices of *ℜ*_0_^*r*^.

Sensitivity index	Sensitivity indices
SI(*β*_2_)	+1
SI(*Λ*)	+1
SI(*σ*)	-0.86
SI(*μ*)	-0.34

## Data Availability

Data used to support the findings of this study are included in the article.
